# Predicting Protein-Protein Interactions via Random Ferns with Evolutionary Matrix Representation

**DOI:** 10.1155/2022/7191684

**Published:** 2022-02-22

**Authors:** Yang Li, Zheng Wang, Zhu-Hong You, Li-Ping Li, Xuegang Hu

**Affiliations:** ^1^School of Computer Science and Information Engineering, Hefei University of Technology, Hefei 230601, China; ^2^School of Information Engineering, Xijing University, Xi'an 710123, China; ^3^School of Computer Science, Northwestern Polytechnical University, Xi'an Shaanxi 710129, China; ^4^College of Grassland and Environment Sciences, Xinjiang Agricultural University, Urumqi 830052, China

## Abstract

Protein-protein interactions (PPIs) play a crucial role in understanding disease pathogenesis, genetic mechanisms, guiding drug design, and other biochemical processes, thus, the identification of PPIs is of great importance. With the rapid development of high-throughput sequencing technology, a large amount of PPIs sequence data has been accumulated. Researchers have designed many experimental methods to detect PPIs by using these sequence data, hence, the prediction of PPIs has become a research hotspot in proteomics. However, since traditional experimental methods are both time-consuming and costly, it is difficult to analyze and predict the massive amount of PPI data quickly and accurately. To address these issues, many computational systems employing machine learning knowledge were widely applied to PPIs prediction, thereby improving the overall recognition rate. In this paper, a novel and efficient computational technology is presented to implement a protein interaction prediction system using only protein sequence information. First, the Position-Specific Iterated Basic Local Alignment Search Tool (PSI-BLAST) was employed to generate a position-specific scoring matrix (PSSM) containing protein evolutionary information from the initial protein sequence. Second, we used a novel data processing feature representation scheme, MatFLDA, to extract the essential information of PSSM for protein sequences and obtained five training and five testing datasets by adopting a five-fold cross-validation method. Finally, the random fern (RFs) classifier was employed to infer the interactions among proteins, and a model called MatFLDA_RFs was developed. The proposed MatFLDA_RFs model achieved good prediction performance with 95.03% average accuracy on *Yeast* dataset and 85.35% average accuracy on *H. pylori* dataset, which effectively outperformed other existing computational methods. The experimental results indicate that the proposed method is capable of yielding better prediction results of PPIs, which provides an effective tool for the detection of new PPIs and the in-depth study of proteomics. Finally, we also developed a web server for the proposed model to predict protein-protein interactions, which is freely accessible online at http://120.77.11.78:5001/webserver/MatFLDA_RFs.

## 1. Introduction

Recognition of protein-protein interactions (PPIs) is distinctly important for understanding various cellular biological activities [1]. The knowledge of PPIs can help us to explore and elucidate the functions of proteins, drug design, new drug development, and the mechanisms of biological activity and related proteins in cells [2]. Additionally, it can also provide new ideas for other studies, such as the ranking of disease genes [3], functional module identification [4], and human disease prevention and treatment. In general, the research approaches for PPIs mainly include two categories: computational-based methods and biological experimental-based methods. In the last decades, many different experimental techniques have been used for large-scale PPIs validation, such as yeast two-hybrid (Y2H) screens [5], coimmunoprecipitation (Co-IP) [6], nuclear magnetic resonance (NMR) [7], protein chip [8], and other high-throughput biological techniques. However, there are some inevitable disadvantages of these methods: they are not only time-consuming and expensive but also suffer from high false-positive rates and weak generalization ability. Thus, it has great practical significance to develop a new effective machine learning approach for PPIs prediction in order to save cost and time, thereby ultimately improving the prediction accuracy of protein interactions. To date, numerous computational approaches have been suggested to detect PPIs based on different data types, including protein domains, genomic information, evolutionary knowledge, structure information, gene fusion, and phylogenetic profiles [9–14]. Although these methods can be used to detect PPIs, the abovementioned methods are not universally applicable unless prior knowledge of the protein is known. Although amino acid sequence information is readily available for a large number of proteins, the 3D structural information of many proteins is still unclear, and the known and available PPIs for most species are still incomplete or very sparse. Consequently, it is particularly important to design novel computational methods for PPI prediction utilizing only protein amino acid sequence information, so as to better employ these abundant protein sequence data.

Numerous previous works have shown that using protein amino acid sequence information alone is sufficient to predict PPIs. So far, many different computational methods based on sequence information have been presented to implement this pattern in PPI prediction, such as combining average blocks with relevance vector machine [15], combining principal component analysis with ensemble extreme learning machine [16], combining conventional auto covariance with support vector machine [17], local descriptors using k-nearest neighbor [18], discrete cosine transformation using weighted sparse representation model [19], and so on. In 2017, Wang et al. [20] proposed a PCVMZM method based on protein sequence. The Zernike moments (ZM) are used as the feature extraction method. ZM can capture multiangle useful and representative information. Probabilistic classification vector machines (PCVM) are a sparse classification model that optimizes the kernel parameters by the expectation-maximization (EM) algorithm, which not only improves the prediction performance of PPIs but also reduces the computational time in the testing phase. The average prediction accuracy achieved by the PCVMZM method was 94.48% on the *Yeast* dataset. In the same year, Du et al. [21] proposed a method called DeepPPI from the angle of deep learning technology by using amphiphilic pseudo amino acid composition feature extraction algorithm to extract features from amino acid sequences, which opens a new way for studying PPIs. This DeepPPI method reached a prediction accuracy of 94.43% on the Saccharomyces cerevisiae dataset. In 2018, Göktepe and Kodaz [22] applied a new technique called weighted skip-sequential conjoint triads to predict PPIs. The method adopts principal component analysis (PCA) to remove noise information, captures protein sequence information by combining Bi-gram representation and Pseudo-amino acid composition, and finally uses support vector machine (SVM) as a prediction classifier to identify interactions between proteins. In the same year, Song et al. [23] presented a novel feature fusion scheme based on random projection ensemble method, which separately used three algorithms (fast fourier transform, discrete cosine transform, and singular value decomposition) to explore and denote the patterns of interactions between amino acids. In 2019, Chen et al. [1] developed an end-to-end framework, called PIPR, to predict PPIs using only the protein sequences. They capture effectively the local significant features and sequential features from protein sequence pairs by using a deep residual recurrent convolutional neural network. Experimental results demonstrate that the framework has good scalability on different datasets. In the same year, Beltran et al. [24] used five feature extraction methods, namely, dipeptide composition, tripeptide composition, autocovariance, amino acid composition, and pseudo-amino-acid composition to represent amino acid sequences. They then employed SVM, random forest (RF), and extreme gradient boosting (XGBoost) to predict PPIs, respectively, and finally achieved good prediction performance. More recently, Jha and Saha [25] presented a deep-learning-based predictor to identify PPIs. They introduced two deep learning algorithms, ResNet50 and stacked autoencoder, to extract features from the autocovariance and conjoint triad representations of protein sequences. Then, LSTM-based classifier model was constructed for each feature encoding scheme. The experimental results show that the introduced deep learning scheme can learn valuable features from multimodal information of proteins. Although a number of computational-based methods have achieved good progress and application prospects, the accuracy and efficiency of PPIs prediction still need to be further enhanced so as to provide a supplementary tool for proteomics research and other bioinformatics tasks.

In this paper, an efficient computational method for detecting PPIs from amino acid sequences is presented by using the evolutionary matrix representation of protein sequences and combining with an ensemble classifier. Among them, an important improvement of the proposed model is to develop a more accurate numerical representation of protein sequences. Specifically, we applied the MatFLDA feature extraction algorithm to a position-specific scoring matrix (PSSM) to extract the evolutionary information of protein sequences and utilized a random ferns classifier to predict the PPIs. More specifically, each protein sequence is denoted as a PSSM numerical matrix. Subsequently, for the purpose of obtaining more representative information, we utilize the MatFLDA descriptor to extract the feature information in each PSSM, so as to obtain a 400-dimensional feature vector from the model and thus obtain an 800-dimensional feature vector representation of each protein pair. Finally, we employ the feature vector of protein pairs as the input of the model and combine the RF ensemble model in machine learning to accomplish the classification task of PPIs. The proposed method is estimated on the PPI datasets of *Yeast* and *H. pylori* with prediction accuracy of 95.03% and 85.35%, respectively. By comparing with a series of previous computational methods, we clearly found that the proposed model has good generalization performance in predicting PPIs.

## 2. Materials and Methodology

### 2.1. Datasets

So far, a number of PPIs databases have been created, including HAPPI database [26], Molecular Interaction Database (MINT) [27], APID database [28], Biomolecular Interaction Network Database (BIND) [29], and Database of Interacting Proteins (DIP) [30]. In this section, we use two high-quality benchmark datasets, which are extracted from DIP, to test the generality of the model and assess the performance of the proposed method. The first dataset is the *yeast* dataset collected by Guo et al. [17]. To evaluate our method, a data preprocessing procedure that deleted protein pairs of greater than 40% sequence identity and less than 50 residues was used in this experiment to avoid the bias introduced by these homologous sequence pairs. By performing this process, we extracted 5594 protein pairs which formed the golden standard positive dataset. The additional 5594 protein pairs were retained to construct the golden standard negative dataset by removing interaction pairs with the same subcellular localization information. The second dataset is the *H. pylori* dataset, which was validated by the yeast two-hybrid technology [31] and collected by Martin et al. [32]. The PPI dataset of *H. pylori* contains 1458 positive protein pairs and 1458 negative protein pairs, which are regarded as positive and negative datasets, respectively. Consequently, *yeast* and *H. pylori* datasets are composed of a total of 11,188 and 2916 protein pairs, respectively.

### 2.2. Numerical Characterization of Protein Sequences

Position-Specific Scoring Matrix (PSSM) serves as a very useful scoring matrix that can contain evolutionary information of protein sequences, which is crucial in proteomics. PSSM was originally introduced by Gribskov et al. [33] in 1987 and is commonly used to detect distantly related proteins and protein folding patterns [34]. Currently, some researchers have done a lot of related work using PSSM encoding information in many fields of bioinformatics such as identification of DNA binding proteins [35], the identification of drug-target interaction [36], prediction of membrane protein types [37], and protein-protein interaction site prediction [38]. In this experiment, we employed the Position-Specific Iterated Basic Local Alignment Search Tool (PSI-BLAST) [39] to convert each protein sequence into a PSSM, which is widely adopted for the numerical representation of protein sequences for further use in PPI detection tasks. PSSM is a matrix composed of *T* rows and 20 columns, where the row represents the length of the protein sequence and 20 columns are attributed to the 20 naive amino acids. Suppose that *M* = {*∂*_*i*,*j*_ : *i* = 1, ⋯, *T* and *j* = 1, ⋯, 20}, PSSM can be described as follows:

(1) $$\begin{array}{c} M=\left[\begin{array}{cccc} \partial_{1,1} & \partial_{1,2} & \cdots & \partial_{1,20}\\ \partial_{2,1} & \partial_{2,2} & \cdots & \partial_{2,20}\\ \vdots & \vdots & \vdots & \vdots \\ \partial_{T,1} & \partial_{T,2} & \cdots & \partial_{T,20} \end{array}\right]. \end{array}$$

The elements in this matrix usually contain positive or negative integers, where the element *∂*_*i*,*j*_ is the probability that the *i*th amino acid mutates into the *j*th amino acid in the process of biological evolution. Here, positive scores in this matrix mean that amino acid substitutions occur more frequently in the alignment, whereas negative scores mean that the substitution occurs less frequently.

In our study, we set the *e*-value and iteration times of PSI-BLAST, which are 0.001 and 3, respectively, to obtain highly and broadly homologous protein sequences. Consequently, each protein sequence is denoted as a 20-dimensional matrix containing *T* × 20 elements, where *T* is the length of a given protein sequence and 20 indicates the number of amino acids. The application information of PSI-BLAST can be downloaded at http://blast.ncbi.nlm.nih.gov/Blast.cgi [40, 41].

### 2.3. Matrix Fisher Linear Discriminant Analysis (MatFLDA)

Fisher linear discriminant analysis (FLDA), as a popular feature extraction method [42], has recently gained considerable attention in the areas of data mining and pattern recognition, such as software fault prediction [43], Arabic text classification [44], and face recognition [45]. In Section 2.2, each PSSM can be denoted as *M* = {*∂*_*i*,*j*_ : *i* = 1, ⋯, *T* and *j* = 1, ⋯, 20}, which is a *T* × 20 matrix. To construct the FLDA of the matrix pattern, we give the matrix pattern *A*_*ij*_ for the *i*th class containing *N*_*i*_ samples, which can be denoted as *A*_*i*j_ = *M*^*T*^ × *M*(*i* = 1, 2, ⋯, *C*, *j* = 1, 2, ⋯, *N*_*i*_), where represents the number of PSSMs, and the total sample mean is defined as $\bar{A}.$ For Matrix Fisher Linear Discriminant Analysis (MatFLDA), assume that a class matrix pattern *A*_*i*_, *i* = 1, 2, ⋯, *C* containing *C* classes is given, where *C* = 20 represents the 20 classes of amino acids, and their class mean is $\bar{A_{i}}.$ Let *x* be a vector with m components. MatFLDA aims to project a matrix pattern *A* onto the *x* satisfying the constraint that *x*^*T*^*x* = 1, and then a 1 × *n* dimensional feature matrix can be generated by using the following linear transformation.

(2) $$\begin{array}{c} y=x^{T}A, \end{array}$$

where *y* is an extracted feature matrix or projected value. Hence, for each matrix pattern *A*_*ij*_, all their feature matrices are projected as follows:

(3) $$\begin{array}{c} y_{ij}=x^{T}A_{ij},i=1,2,\cdots ,C;j=1,2,\cdots ,N_{i}. \end{array}$$

To find the optimal projection vector *x*, we use the following criterion function and maximize it:

(4) $$\begin{array}{c} J_{Mat}\left(x\right)=\frac{tr\left(x^{T}S_{b}^{Mat}x\right)}{tr\left(x^{T}S_{w}^{Mat}x\right)}, \end{array}$$

where *S*_*b*_^*Mat*^ is the total between-class scatter matrix, which is defined as

(5) $$\begin{array}{c} S_{b}^{Mat}=\overset{C}{\underset{i=1}{\sum }}N_{i}\left(\bar{A_{i}}-\bar{A}\right){\left(\bar{A_{i}}-\bar{A}\right)}^{T}, \end{array}$$

where *S*_*w*_^*Mat*^ is the total within-class scatter matrix, which is defined as

(6) $$\begin{array}{c} S_{w}^{Mat}=\overset{C}{\underset{i=1}{\sum }}\overset{N_{i}}{\underset{j=1}{\sum }}\left(A_{ij}-\bar{A_{i}}\right){\left(A_{ij}-\bar{A_{i}}\right)}^{T}. \end{array}$$

In the MatFLDA algorithm, by maximizing *J*_*Mat*_(*x*), we want to keep the between-class scatter matrix as large as possible and the within-class scatter matrix as small as possible in the projection space. Furthermore, under the constraint *x*^*T*^*x* = 1, this optimization problem can be further equated to solve the following eigenvalue-eigenvector matrix equation:

(7) $$\begin{array}{c} S_{b}^{Mat}x=\lambda S_{w}^{Mat}x. \end{array}$$

At last, the completely new features are obtained by determining the appropriate *x*, which will be used in the subsequent classification task. In this experiment, the PSSM of *N* protein sequences of size *T* × 20 was used as input to the Matflda algorithm on the *yeast* and *H. pylori* datasets, where the Matflda algorithm was only used for feature extraction. In this way, we obtained the output of a 20 × 20 dimensional feature matrix by using the MatFLDA algorithm on an original PSSM of protein sequence. In other words, we obtained a feature vector of 1 × 400 dimensions from each PSSM. Consequently, the output of *N* PSSMs is *N* fixed size 20 × 20 dimensional feature matrices. Thus, each protein pair contains 800 features. Here, in order to clearly understand how to use the MatFLDA algorithm for feature extraction of protein sequences, we give a schematic diagram of MatFLDA feature extraction for a protein pair namely Histone H4 and Regulatory protein SIR3 in the *Saccharomyces cerevisiae* dataset, as shown in Figure 1.

### 2.4. Random Ferns (RFs)

Random fern classifier is developed based on random forests, but it is different from the random forest [46, 47]. Here, by giving a PSSM in a protein sequence, our main task is to assign it to the most likely class. Let *c*_*i*_, *i* = 1, 2, be the set of classes, where 1 indicates an interacting protein and 2 is a noninteracting protein. Let *x*_*j*_, *j* = 1, 2, ⋯, *N*, be the set of normalized 20 × 20 dimensional features that will be calculated by using the MatFLDA algorithm on the PSSM that we are trying to classify. Formally, we are looking for [48]

(8) $$\begin{array}{c} {c_{i}}^{\prime }=\underset{c_{i}}{\arg\max}\;P\left(\left.C=c_{i}\right|x_{1},x_{2},\cdots ,x_{N}\right), \end{array}$$

where *C*, a random variable, represents the class of protein. The aim of this paper is to model the posterior interacting protein class probability by giving a set of *N* features. This can be expressed in terms of the Bayesian formula, as

(9) $$\begin{array}{c} P\left(\left.C=c_{i}\right|x_{1},x_{2},\cdots ,x_{N}\right)=\frac{P\left(\left.x_{1},x_{2},\cdots ,x_{N}\right|C=c_{i}\right)\times P\left(C=c_{i}\right)}{P\left(x_{1},x_{2},\cdots ,x_{N}\right)}. \end{array}$$

Assuming a uniform prior *P*(*C*), since the denominator is just a scale factor, it is independent and is common for all the classes. Thus, by removing the priors *P*(*x*_1_, *x*_2_, ⋯, *x*_*N*_), the problem reduces to finding

(10) $$\begin{array}{c} {c_{i}}^{\prime }=\underset{c_{i}}{\arg\max}\;P\left(\left.x_{1},x_{2},\cdots ,x_{N}\right|C=c_{i}\right). \end{array}$$

But learning the complete representation of the joint probability of all features is very intractable. According to the Naive Bayes theory, it is assumed that all features are completely independent, that is,

(11) $$\begin{array}{c} P\left(\left.x_{1},x_{2},\cdots ,x_{N}\right|C=c_{i}\right)=\overset{N}{\underset{j=1}{\prod }}P\left(\left.x_{j}\right|C=c_{i}\right). \end{array}$$

However, this independence assumption is usually wrong because it completely ignores the correlation between features in practice. To account for the dependencies between these features while making the problem tractable, a better compromise is to divide our features into *M* groups of size *S* = *N*/*M*. These groups are what we define as ferns, and we calculate the joint probability for features in each fern. The conditional probability is expressed as follows:

(12) $$\begin{array}{c} P\left(\left.x_{1},x_{2},\cdots ,x_{N}\right|C=c_{i}\right)=\overset{M}{\underset{k=1}{\prod }}P\left(\left.F_{k}\right|C=c_{i}\right). \end{array}$$

where *F*_*k*_ = {*x*_*ϑ*(*k*, 1)_, *x*_*ϑ*(*k*, 2)_, ⋯, *x*_*ϑ*(*k*, *S*)_}, *k* = 1, ⋯, *M*, refers to the *k*th fern, and *ϑ*(*k*, *j*) is a random permutation function. Therefore, we follow a seminaive Bayesian method by modeling only some of the dependencies between features. In addition, the class conditional probabilities *P*(*F*_*m*_|*C* = *c*_*i*_) are estimated for each fern *F*_*m*_ and class *c*_*i*_ in the training phase. For each fern *F*_*m*_, these terms can be described as

(13) $$\begin{array}{c} p_{k,c_{i}}=P\left(F_{m}=k\;|\;C=c_{i}\right)=\frac{N_{k,c_{i}}}{N_{c_{i}}}, \end{array}$$

where *N*_*k*,*c*_*i*__ represents the number of training samples of class *c*_*i*_ that evaluates to fern value *k*, *k* = 1, 2, ⋯, *K*. Here, *K* = 2^*S*^, and *N*_*c*_*i*__ represents the total number of samples for class *c*_*i*_. However, when the number of samples given is not infinitely large, both *N*_*k*,*c*_*i*__ and *p*_*k*,*c*_*i*__ will be zero. To overcome this problem, *p*_*k*,*c*_*i*__ is rewritten as

(14) $$\begin{array}{c} p_{k,c_{i}}=\frac{N_{k,c_{i}}+N_{r}}{N_{c_{i}}+K\times N_{r}}, \end{array}$$

where *N*_*r*_ is a regularization term, which behaves as a uniform Dirichlet prior over feature values. *N*_*r*_ = 1 is used to guarantee the results above zero. In this experiment, we set two important parameters of the random ferns classifier, where *S* (the depth of ferns) was set to 20 and *M* (the number of ferns) was set to 140. Finally, the features extracted by the MatFLDA algorithm are normalized and then fed into the random ferns classifier to predict whether each protein pair interacts with each other.

## 3. Results and Discussion

### 3.1. Evaluation Criteria

In this paper, to ensure the robustness of the proposed model and avoid overfitting and data dependency, we adopted five-fold cross-validation to assess the effectiveness of this method in predicting PPIs. Specifically, we first divide the experimental dataset into five parts and then select four of them as the training dataset and the additional one as the testing dataset. Finally, the average values of the five independent experiments are used as prediction results. Here, the following assessments are used, including overall prediction accuracy (ACC), precision (PE), sensitivity (SN), and Matthews correlation coefficient (MCC), which are defined as follows

(15) $$\begin{array}{c} \text{ACC}=\frac{\text{TP}+\text{TN}}{\text{TP}+\text{TN}+\text{FP}+\text{FN}}, \end{array}$$

(16) $$\begin{array}{c} \text{PE}=\frac{\text{TP}}{\text{TP}+\text{FP}}, \end{array}$$

(17) $$\begin{array}{c} \text{SN}=\frac{\text{TP}}{\text{TP}+\text{FN}}, \end{array}$$

(18) $$\begin{array}{c} \text{MCC}=\frac{\text{TP}\times \text{TN}‐\text{FP}\times \text{FN}}{\sqrt{\left(\text{TP}+\text{FP}\right)\left(\text{TP}+\text{FN}\right)\left(\text{TN}+\text{FP}\right)\left(\text{TN}+\text{FN}\right)}}, \end{array}$$

where TP, TN, FP, and FN represent true positive, true negative, false positive, and false negative, respectively. Among them, TP indicates the number of true PPIs that are predicted correctly, TN represents the number of true noninteracting pairs that are predicted correctly. FP indicates the number of true interacting pairs not found in positive dataset, and FN represents the number of true interacting pairs not found in negative dataset. MCC is used as a balance indicator to measure the quality of binary classification in data mining, which value ranges between -1 and +1 representing the correlation coefficient between the observed results and the predicted results. In this experiment, the receiver operating characteristic (ROC) curve [49] and the area under the ROC curve (AUC) [50] are employed to evaluate the prediction performance of the proposed model. The AUC value of the classifier is larger, the prediction performance of the method is superior, and the model constructed is more stable. The flow of the proposed scheme is shown in Figure 2.

### 3.2. Prediction Performance of Proposed Model

In order to assess the effectiveness and stability of the model combining MatFLDA and RFs to predict PPIs, we tested the model on *Yeast* and *H. pylori* datasets in this section. In addition, for reducing deviations of the proposed method and avoiding overfitting, five-fold cross-validation was performed in the experiment. Specifically, the whole dataset was divided into five parts, including five training and five testing datasets, respectively, and then we obtained five models by carrying out separate experiments for each dataset. Finally, the average values of the five models were selected as the prediction results of our experiments. In order to obtain more accurate and reliable experimental results, the fern size *S* and fern number *M* of the random ferns classifier were set to be the same on *Yeast* and *H. pylori* datasets. Here, *S* = 20 and *M* = 140. The five-fold cross-validation prediction results of the RFs prediction model employing the MatFLDA feature extraction algorithm of protein sequence on two benchmark datasets are shown in Tables 1 and 2.

As can be seen from Table 1, the accuracies of the five experiments were 95.26%, 94.99%, 94.81%, 94.77%, and 95.31% when PPIs were performed on the *Yeast* dataset. The precisions are ≥98.81%, the sensitivities are ≥90.27%, and the MCCs are ≥90.05%. The standard deviations corresponding to these four assessment values are 0.25%, 0.26%, 0.47%, and 0.45%, respectively. At the same time, we can see that these standard deviations are relatively low. Similarly, the average values of accuracy, precision, sensitivity, and MCC were 85.35%, 79.27%, 95.72%, and 74.41% when exploring PPIs of *H. pylori* dataset. We can see from Table 2 that the standard deviations corresponding to these four evaluation values are 0.64%, 0.81%, 0.92%, and 1.14%, respectively. In order to better visualize the performance of combining RFs and MatFLDA to predict PPIs, we plot the ROC curves on two benchmark datasets. In addition, MCC and AUC values were also calculated to better quantify the predictive performance of the proposed model. The ROC curves performed on the two benchmark datasets are shown in Figures 3 and 4.

From Figures 1 and 2, we can see that the average AUC values obtained by the proposed method were 94.27% and 94.12% for the experiments on *Yeast* and *H. pylori* datasets, respectively. The promising results show that the proposed method is feasible, effective, and practical for detecting PPIs. The excellent prediction performance mainly depends on the selection of the feature extraction algorithm and classification model of the proposed method. It can be seen that the MatFLDA feature extraction descriptor can effectively retain useful information from the original protein sequences. Moreover, the high prediction accuracies and low standard deviations further indicate that the proposed method is robust for predicting PPIs.

### 3.3. Comparison of the Four Methods Using the Same Feature Representation

Generally, the same feature extraction approach by combining different classifiers will yield different prediction results when using machine-learning-based methods to predict PPIs. In this section, we performed PPI experiments using the same feature extraction method on the state-of-the-art individual classifier support vector machine (SVM) and the proposed ensemble learning classifier random ferns in order to further evaluate the prediction performance of the proposed model. It should be noted that the LIBSVM toolbox, which was downloaded from https://www.csie.ntu.edu.tw/~cjlin/libsvm/ [51], was employed in this experiment to carry out the PPI classification task. In our experiment, a polynomial function is used as the kernel function and the initial values of SVM are *c* = 0.1, *g* = 0.2 and *c* = 0.01, *g* = 0.1 when predicting PPIs using five-fold cross-validation on *Yeast* and *H. pylori* datasets, respectively. For SVM and RF classifiers, all input feature vectors are normalized by the zero-mean normalization method.

The experimental results of PPIs based on RFs and SVM-based classifiers are presented in Tables 3 and 4 on *Yeast* and *H. pylori* datasets, respectively. From Table 3, the average values of accuracy, precision, sensitivity, and MCC of the RF method on *Yeast* dataset are as high as 95.03%, 99.14%, 90.84%, and 90.52%, respectively. However, when employing the SVM classifier, we yielded relatively poor prediction results with the average values of accuracy, precision, sensitivity, and MCC of 80.39%, 83.01%, 76.44%, and 68.38%, respectively. It can be observed that the maximum accuracy obtained by the SVM classifier is 81.63%, which is 13% lower than the minimum accuracy obtained by the RF method. Similarly, as presented in Table 4, the average accuracy by utilizing SVM method in *H. pylori* dataset is 82.09%, among which the results of five models are 82.85%, 82.33%, 79.42%, 82.33%, and 83.53%, respectively. Additionally, for further evaluation, the ROC (receiver operating characteristic) curves and AUC values based on the SVM method are also calculated (see Figures 5 and 6). The average AUC values obtained by the same feature extraction method on *Yeast* and *H. pylori* datasets were 85.78% and 88.94%, respectively. In addition, we also evaluate the prediction performance of the proposed model using Random Forest and XGBoost classifiers by employing the same features. Comparing the proposed model with these three models, we can clearly see the proposed model achieves good performance in the prediction of PPIs. Thus, the proposed model can provide a useful tool for detecting PPIs and other bioinformatics tasks.

### 3.4. Comparison with other PPI Prediction Methods

Currently, many computational methods that are based on data mining knowledge have been presented for predicting sequence-based PPIs. In this section, to verify the performance of the proposed model, we measure the proposed method by comparing with several other state-of-the-art methods on the *Yeast* and *H. pylori* datasets. Specifically, we compared the proposed method with previous work on PPI prediction presented by Guo et al., Yang et al., Zhou et al., You et al., Du et al., and Wong et al. on the *Yeast* dataset.  Table 5 lists the PPI prediction results of the above methods on the same *Yeast* dataset.

As shown in Table 5, the accuracy, sensitivity, precision, and MCC of the MatFLDA_RFs method are 95.03%, 90.84%, 99.14%, and 90.52%, respectively. Compared with other existing methods listed, the accuracy of the proposed method increased by about 0.1% to 9%. The ACC of MatFLDA_RFs method is 7.67% higher than the AC method, 8.88% higher than the Cod4 + KNN method, 6.47% higher than the SVM + LD method, 3.67% higher than the MCD + SVM method, 0.89% higher than the LRA + RF method, 0.60% higher than the DeepPPI method, and 1.11% higher than the PR − LPQ + RF method. The PE of MatFLDA_RF method is 11.32% higher than the AC method, 8.90% higher than the Cod4 + KNN method, 9.64% higher than the SVM + LD method, 7.20% higher than the MCD + SVM method, 2.04% higher than the LRA + RF method, 2.49% higher than the DeepPPI method, and 2.69% higher than the PR − LPQ + RF method. The MCC of MatFLDA_RFs method is 13.37% higher than the SVM + LD method, 6.31% higher than the MCD + SVM method, 1.56% higher than the LRA + RF method, 1.55% higher than the DeepPPI method, and 1.96% higher than the PR − LPQ + RF method.

Similarly, Table 6 presents the PPI prediction results of other existing methods on the same *H. pylori* dataset. As shown in Table 6, the prediction performance of the proposed method is better than other existing methods. The obtained values of ACC, SN, PE, and MCC are 85.35%, 95.72%, 79.27%, and 74.41%, respectively. In terms of ACC, the MatFLDA_RFs method is 0.44%-9.55% higher than other methods, 1.95% higher than the Signature Products + SVM method, 0.44% higher than the MCD + SVM method, 1.65% higher than the WSR method, 9.55% higher than the Phylogenetic Booststrap method, 2.35% higher than the LDC method, and 5.83% higher than the Boosting method. These excellent results prove that the proposed method is an effective computational tool suitable for predicting PPIs.

## 4. Conclusion

The study of proteins and their interactions is essential to understand most biological activities in living cells, such as development, signal transduction, and apoptosis. Therefore, the successful prediction of PPIs will facilitate the study of other related problems in biomedical science. In this work, we present a novel computational approach to detect PPIs, using the MatFLDA algorithm, the RF classifier, and the PSSM matrix that can preserve protein evolutionary information. More specifically, MatFLDA is used to obtain the feature representation from the PSSM, an evolutionary matrix of protein sequences. This PSSM contains a great deal of valuable and important knowledge for PPI prediction. The RF classifier is then applied to detect novel PPIs. Finally, to measure the PPI identification ability of the developed method, we conducted extensive computational experiments on several benchmark PPI datasets. These excellent experimental results have indicated that the proposed MatFLDA_RF method has a higher identification rate of PPIs than other existing methods and SVM-based approaches. Consequently, the proposed method to identify PPIs is reliable and effective, which can be used as a practical tool for experimental methods, thus, facilitating further research on related problems in the field of bioinformatics.

## Figures and Tables

**Figure 1:** Flow chart of MatFLDA feature extraction for each protein pair.

**Figure 2:** The flow of the proposed scheme.

**Figure 3:** ROC curves performed using the proposed method on *Yeast* dataset.

**Figure 4:** ROC curves performed using the proposed method on *H. pylori* dataset.

**Figure 5:** ROC curves performed using the SVM method on *Yeast* dataset.

**Figure 6:** ROC curves performed using the SVM method on *H. pylori* dataset.

**Table 1:** Five-fold cross-validation prediction results achieved in predicting *Yeast* PPI dataset.

Testing set	ACC (%)	PE (%)	SN (%)	MCC (%)	AUC (%)
1	95.26	99.41	91.06	90.94	94.79
2	94.99	99.33	90.85	90.47	93.44
3	94.81	98.81	90.55	90.12	94.11
4	94.77	99.21	90.27	90.05	94.00
5	95.31	98.92	91.49	91.02	94.99
Average	95.03 ± 0.25	99.14 ± 0.26	90.84 ± 0.47	90.52 ± 0.45	94.27 ± 0.63

**Table 2:** Five-fold cross-validation prediction results achieved in predicting *H. pylori* PPI dataset.

Testing set	ACC (%)	PE (%)	SN (%)	MCC (%)	AUC (%)
1	85.76	79.30	95.77	75.19	94.16
2	85.59	79.15	96.56	74.76	93.63
3	85.59	79.27	94.20	75.11	94.28
4	85.59	80.44	95.74	74.58	93.78
5	84.22	78.17	96.35	72.43	94.78
Average	85.35 ± 0.64	79.27 ± 0.81	95.72 ± 0.92	74.41 ± 1.14	94.12 ± 0.45

**Table 3:** Five-fold cross-validation results by using two models on the *Yeast* dataset.

Classifier	Testing set	ACC (%)	PE (%)	SN (%)	MCC (%)	AUC (%)
SVM	1	81.63	84.29	77.73	69.91	87.06
	2	80.02	83.86	75.61	67.92	86.23
	3	79.44	80.79	76.39	67.25	84.55
	4	80.20	83.28	75.63	68.11	84.74
	5	80.69	82.83	76.83	68.72	86.34
	Average	80.39 ± 0.82	83.01 ± 1.36	76.44 ± 0.89	68.38 ± 1.00	85.78 ± 1.09
RFs	1	95.26	99.41	91.06	90.94	94.79
	2	94.99	99.33	90.85	90.47	93.44
	3	94.81	98.81	90.55	90.12	94.11
	4	94.77	99.21	90.27	90.05	94.00
	5	95.31	98.92	91.49	91.02	94.99
	Average	95.03 ± 0.25	99.14 ± 0.26	90.84 ± 0.47	90.52 ± 0.45	94.27 ± 0.63
Random Forest	Average	95.48 ± 0.29	97.71 ± 0.38	93.14 ± 0.71	91.35 ± 0.53	95.48 ± 0.28
XGBoost	Average	94.08 ± 1.08	96.43 ± 0.92	91.54 ± 1.52	88.86 ± 1.91	98.59 ± 0.34

**Table 4:** Five-fold cross-validation results by using two models on the *H. pylori* dataset.

Classifier	Testing set	ACC (%)	PE (%)	SN (%)	MCC (%)	AUC (%)
SVM	1	82.85	81.72	83.45	71.57	89.26
	2	82.33	80.52	85.22	70.86	89.87
	3	79.42	76.17	82.25	67.25	86.20
	4	82.33	83.22	82.95	70.85	89.16
	5	83.53	84.75	83.06	72.47	90.22
	Average	82.09 ± 1.57	81.28 ± 3.26	83.39 ± 1.12	70.60 ± 1.99	88.94 ± 1.60
RFs	1	85.76	79.30	95.77	75.19	94.16
	2	85.59	79.15	96.56	74.76	93.63
	3	85.59	79.27	94.20	75.11	94.28
	4	85.59	80.44	95.74	74.58	93.78
	5	84.22	78.17	96.35	72.43	94.78
	Average	85.35 ± 0.64	79.27 ± 0.81	95.72 ± 0.92	74.41 ± 1.14	94.12 ± 0.45
Random Forest	Average	87.27 ± 0.82	85.90 ± 0.72	89.09 ± 2.45	77.73 ± 1.21	93.28 ± 0.69
XGBoost	Average	85.11 ± 1.22	84.28 ± 3.10	86.49 ± 3.25	74.64 ± 1.72	91.59 ± 0.82

**Table 5:** The prediction ability of the other methods on the *Yeast* dataset.

Related work	Method	ACC (%)	SN (%)	PE (%)	MCC (%)	AUC (%)
Guo et al.'s work [17]	AC	87.36 ± 1.38	87.30 ± 4.68	87.82 ± 4.33	N/A	N/A
	ACC	89.33 ± 2.67	89.93 ± 3.68	88.87 ± 6.16	N/A	N/A
Yang et al.'s work [18]	Cod4 + KNN	86.15 ± 1.17	81.03 ± 1.74	90.24 ± 1.34	N/A	N/A
Zhou et al.'s work [52]	SVM + LD	88.56 ± 0.33	87.37 ± 0.22	89.50 ± 0.60	77.15 ± 0.68	95.07 ± 0.39
You et al.'s work [53]	MCD + SVM	91.36 ± 0.36	90.67 ± 0.69	91.94 ± 0.62	84.21 ± 0.59	97.07 ± 0.12
You et al.'s work [54]	LRA + RF	94.14 ± 1.8	91.22 ± 1.6	97.10 ± 2.1	88.96 ± 2.6	94.20 ± 1.7
Du et al.'s work [21]	DeepPPI	94.43 ± 0.30	92.06 ± 0.36	96.65 ± 0.59	88.97 ± 0.62	N/A
Wong et al.'s work [55]	PR − LPQ + RF	93.92 ± 0.36	91.10 ± 0.31	96.45 ± 0.45	88.56 ± 0.63	N/A
Proposed method	MatFLDA_RFs	95.03 ± 0.25	90.84 ± 0.47	99.14 ± 0.26	90.52 ± 0.45	94.27 ± 0.63

Note: N/A means not available.

**Table 6:** The prediction ability of the different methods on the *H. pylori* PPI dataset.

Related work	Method	ACC (%)	SN (%)	PE (%)	MCC (%)
Martin et al.'s work [32]	Signature products + SVM	83.40	79.90	85.70	N/A
You et al.'s work [53]	MCD + SVM	84.91	83.24	86.12	74.40
Nanni's work [56]	WSR	83.70	79.00	87.00	N/A
Bock and Gough's work [57]	Phylogenetic Booststrap	75.80	69.80	80.20	N/A
Nanni's work [56]	LDC	83.00	80.60	85.10	N/A
Shi et al.'s work [58]	Boosting	79.52	80.37	81.69	70.64
Proposed method	MatFLDA_RFs	85.35	95.72	79.27	74.41

Note: N/A means not available.

## Data Availability

The data used to support the findings of this study are available from the corresponding author upon request.
